# A Systematic Review on Antimicrobial and Antiparasitic Activity of *Eurycoma longifolia* Jack (Tongkat Ali)

**DOI:** 10.1155/2022/4999797

**Published:** 2022-07-06

**Authors:** Mohd Qayyum Ab Latip, Mohd Hezmee Mohd Noor, Hafandi Ahmad, Hasliza Abu Hassim, Annas Salleh, Mohd Hair Bejo, Alif Aiman Zakaria

**Affiliations:** ^1^Department of Veterinary Preclinical Sciences, Faculty of Veterinary Medicine, Universiti Putra Malaysia, 43400 Serdang, Selangor, Malaysia; ^2^Department of Veterinary Pathology and Microbiology, Faculty of Veterinary Medicine, Universiti Putra Malaysia, 43400 Serdang, Selangor, Malaysia

## Abstract

*Eurycoma longifolia* or Tongkat Ali (family: Simaroubaceae) has the potential to be utilised as an antimicrobial and antiparasitic agent that correlated with its traditional use to treat jaundice, malaria, antiseptic agent, and many more. This review is aimed at systematically sieving through articles regarding the antimicrobial and antiparasitic activity of *E. longifolia*. A total of 123 studies have been found using suitable keywords and manually searched from previous studies through the four databases. After title screening and abstract examination, 56 articles were excluded due to duplication and not meeting the acceptance criteria. 67 articles were assessed on full-text accessibility, 31 studies remained, and this number decreased to 20 articles after a careful examination of the full-text articles. Among the 20 articles selected, 17 articles proved the potential of *E. longifolia* as an antimicrobial and antiparasitic agent efficiently. 2 selected articles showed partial positive results, which specified specific microorganisms tested. In contrast, another 1 article gave a completely negative result. As for the conclusion, current studies highlighted by this review may shed light on the future direction of studies concerning *E. longifolia* as a novel antimicrobial and antiparasitic agent. However, more research should be done in the future focusing on the efficiency of *E. longifolia* for veterinary medicine utilisation.

## 1. Introduction

Antimicrobials are compounds that are active against microorganisms, which include bacteria and fungi. Their mode of action either inhibits microorganisms' growth or destroys them completely. Due to its efficiency in curing infection, antimicrobial drugs were hugely consumed, especially in veterinary medicine. Not just treatment, the need for antimicrobials is also heavily influenced by husbandry practices that directly link to animal health. Mackinnon [1] stated that the use of prophylactic antibiotics through intramammary infusion can be effective at the end of the lactation period as a prevention step of dry period intramammary infection in dairy cows.

Currently, antimicrobial resistance is a worldwide issue, as it becomes a major public health concern globally. It does not just focus on the human basis, but research has rooted it down to its potential sources. Despite uncontrollable consumption of drug descriptions, daily intake of food sources is also being considered. Consumption of livestock treated with the antimicrobial drug particularly worried us even though it was under strict quality control. Based on Woolhouse et al. [2], although the usage of growth promoters using antibiotics had been banned, antibiotic usage still has not consistently decreased.

Antimicrobial drugs are an important part of veterinary medicine because they can enhance animal health and production, as well as contribute to food safety, food security, livelihood protection, animal resource protection, and animal welfare. However, the risk of antimicrobial resistance should be identified and discussed. Clear policy issues and knowledge gaps in monitoring antimicrobial resistance should be applied. Replacing antimicrobial drugs with natural herbs that mimic the pharmacokinetics of those drugs would be highly benefitted. Perumal Samy and Gopalakrishnakone [3] concluded that traditional plants can be new sources of antimicrobials in modern medicine as their stable biologically active compound can establish a scientific base.

Besides antimicrobial resistance issues, the parasitic disease has become a significant challenge for human well-being and animal basis. One of them was malaria, and it was a serious issue, especially for the poor population, who lived in tropical and subtropical regions with economies that were struggling. Malaria affects more than 500 million people globally each year, resulting in over one million deaths, according to the World Health Organization (WHO). In 2019, 229 million estimated malaria cases were reported worldwide [4]. The suburban region hit the most malaria cases, classified by WHO as a high burden to high impact (HBHI) countries. Malaria is a life-threatening parasitic disease caused by *Plasmodium*. Malaria is spread through bites from infected *Anopheles* mosquitoes, sometimes known as malaria vectors. Due to unaffordable drugs and inaccessible health facilities in particularly suburban areas, the mortality rate had peaked.

Another parasitic disease that currently comes into consent is toxoplasmosis. This disease is caused by infection with the *Toxoplasma gondii* parasite, which is one of the most widespread parasites in the world. In small animal veterinary practices, toxoplasmosis has become a common case diagnosed in veterinary clinics. Mainly, affected cats will have developed fever, loss of appetite, weight loss, lethargy and worse cases, pneumonia, and glaucoma. OIE Terrestrial Manual 2017 stated that toxoplasmosis is a zoonotic disease that affects human health risks. Pregnant women are the most high-risk individuals, which may result in abortion due to the infection. The most likely sources of human infection are exposed to infected cats' faeces and consumption of raw infected meat, which contains live *T. gondii* tissue cysts.

In order to solve these two major issues, potential solutions for future approaches have been identified. The new antimicrobial and antiparasitic medicines with significant clinical findings can be used to address these problems. It is crucial to replace the pharmaceutical pipeline to have better prospects and advanced stages of treatment. The return to the search for natural products is highly recommended. Due to their natural origin, plant extracts are excellent candidates to replace synthetic compounds, which are believed to have carcinogenic and toxicological effects [5].

Since antiquity, herbal and traditional medicine has already been used as a conventional method of improving health. Currently, the medicinal benefits of the herbal plant are being largely explored, especially in pharmacological and toxicological studies. The high amount of biologically active compounds, which have low side effects, is the main reason these researchers have come up with the reverse way of treatment. To introduce the natural products back into the treatment regime, sufficient research and clinical experiment must be conducted to prove the therapeutic effect, especially against microbes and parasites.

In Malaysia, *Eurycoma longifolia* Jack is considered a national treasure which be called as “Tongkat Ali,” while other countries referred it as Malaysian Ginseng. It is a Southeast Asian plant that has been used in traditional medicine for centuries. Since ancient times, people have relied on the medicinal properties of this plant's aqueous decoction. Traditional uses of the plant parts include antimicrobial, antimalarial, antidiabetic, aphrodisiac, antibacterial, and antipyretic properties. Various bioactive components such as eurycomanone, eurycomaside, eurycolactone, eurycomalatone, and pasakbumin-B, in which the quassinoids and alkaloids are a significant portion of the plant parts, make this plant need to be evaluated on its toxicity and safety [6]. Although the traditional practices have shown an effective effect, research on scientific databases of commercial utilisation of Tongkat Ali still needs to be done regarding consumer safety, especially in veterinary medicine practices.

## 2. Methodology

This systematic review was carried out following these five main subsections, namely PRISMA, resources, eligibility and exclusions criteria, systematic review procedure, data abstraction, and analysis, applied in the current research. Then, the retrieved articles were assessed on the risk of bias.

### 2.1. PRISMA

PRISMA (Preferred Reporting Items for Systematic Reviews and Meta-Analyses) is a guideline for systematic literature reviews reporting. Generally, PRISMA provides a straightforward way of describing and reporting the systematic reviews to assess the pros and cons of a health care intervention [7]. Referring to Sierra-Correa and Cantera Kintz [8], three benefits have been promoted: first, it provides understandable research questions needed in systematic research; second, it specifies acceptance and rejection criteria; and third it is ideal for analysing an extensive scientific literature database makes it often utilised within medical studies. Hence, this systematic review of antimicrobial and antiparasitic properties of *E. longifolia* Jack was guided by the PRISMA statement as the review protocol.

### 2.2. Resources

The review methods of the present study relied on four main databases, namely Scopus, Medline (PubMed), ScienceDirect, and Google Scholar. Considering that these databases are reliable and provide full text for thousands of highly ranked medical journals with cover-to-cover indexing, it would best to be utilised efficiently using correct and specific searching terms. For each database, the search method was adjusted accordingly and is listed in Table 1. Suarez-Almazor et al. [9] suggested that a comprehensive search can be obtained through more databases. Therefore, the present study was hand searching manually on several established sources using Google Scholar to increase the likelihood of obtaining relevant articles.

### 2.3. Eligibility and Rejection Criteria

A few criteria for eligibility and rejection are identified. Studies that evaluated the antimicrobial and antiparasitic activities of extracts of *E. longifolia*, with no limitation on study populations, were chosen. The following acceptance criteria were used: About the type of literature, only article journals publishing with empirical data are considered, which were written in English, have timeline indexes between 2001 and 2021, and evaluated *E. longifolia* antimicrobial or antiparasitic activities or both, with a reliable control group. When the control uses more than one (e.g., untreated medium and a commercial reference of antibiotics), the first one will be selected as a control group. As for the rejection criteria, the literature types of a review article, book, book series, chapter in books, and conference proceedings were discarded. Besides, the search effort also excluded non-English publications timeline indexes before 2001, studies unrelated to the assessment of antimicrobial and antiparasitic activities of *E. longifolia* and lacked a control experiment.

### 2.4. Systematic Review Process

In this section, the systematic review process was categorised into four stages. First, keywords that were used in the search process were identified. Depending on previous studies, the similar keywords and related to antimicrobial and antiparasitic activities were used (Table 2). At this phase, by using the duplication detector tool in the Mendeley Desktop, four articles that were duplicated were discarded.

The second phase was screening. The remaining 119 articles were carefully screened based on the abstract provided by the publisher. In this stage, 52 articles had been excluded due to a lack of acceptance criteria and posed the rejection criteria. The remaining 67 articles were carried into the third phase, which is accessibility, where only articles with full-text access were taken. The last phase of the review was eligibility. Only research articles focusing on *E. longifolia* antimicrobial and antiparasitic activities or both, containing suitable empirical data and a clear experiment, were taken.

### 2.5. Data Abstraction and Analysis

The purpose of this study is to evaluate and analyse previous research analyses that have addressed the formulated questions. In order to evaluate suitable themes and subthemes, the data needed to be identified first through the abstract and then through the full articles (in-depth). Data were extracted individually when the research article evaluated more than one plant extract, chemical substance, or antibiotic reference, focusing on *E. longifolia* antimicrobial and antiparasitic activities. Data regarding the experiment were extracted and analysed using Microsoft Office Excel 2016.

The Mixed Method Appraisal Tool (MMAT), version 2018, was used to evaluate the methodological quality for each article. The low methodological quality of articles based on the overall score would be excluded to increase the sensitivity analysis. The overall score was calculated based on the manual guidance [10].

## 3. Results

### 3.1. Study Selection

The recent systematic review flowchart can be found in Figure 1. After the database searching using the keywords stated in Table 1, 123 studies have been identified. The titles were screened, and the abstract was examined carefully. After the screening process and removal of duplication, a total of 67 articles have remained. Full texts of the remaining articles were analysed to determine if they met the criteria for eligibility. Among them, 36 articles were removed because they did not have access to the full text, and 11 were removed because they did not meet the acceptance criteria. In total, 103 studies were removed for the reasons mentioned in Figure 1. After title screening and abstract examination, 56 articles were excluded due to duplication and not meeting the acceptance criteria. 67 articles were assessed on full-text accessibility, 31 articles remained, and the number was decreased to 20 articles after a particular examination through the full text articles; 20 articles were used in this study.

### 3.2. Characteristics of the Included Articles

The characteristics of 20 selected studies are listed in Table 2.

## 4. Discussion

*Eurycoma longifolia* has been shown to be an antimicrobial and antiparasitic agent through this systematic review. This manuscript hypothesised that *E. longifolia* could minimise or inhibit bacterial, fungal, and parasitic growth. From 20 articles, 10 studies evaluated *E. longifolia*'s antimicrobial effects, and another 10 studies evaluated its antiparasitic effects on selected microorganism species (Table 3). Among these studies, 19 of them were in vitro studies, and only 1 in vivo study was managed to include in this review.

In most of these studies, the sample size of the test groups is mostly small. Samples from each group are usually done in triplicates. Additionally, the duration of exposure time for these 20 studies ranges from 22 to 72 hours. It is possible that the research designs used in these experiments have limitations due to these facts.

### 4.1. Effectiveness of Antimicrobial Activity of *E. longifolia*

In 10 in vitro studies for antimicrobial activity that were obtained, 18 microorganisms' species were used in these studies (Table 3). Based on the results, it showed that *E. longifolia* showed antimicrobial activity on most of the microorganisms tested, in which 7 out of 10 studies showed complete positive results. However, 2 of studies ( [14, 17] showed partial positive results that vary among the tested microorganism species and the plant component used. 1 of the study by Yi Xin et al. [29] showed a completely negative result.  Table 4 shows the result extracted from 10 studies which evaluate on antimicrobial activity of *E. longifolia*.

Alloha et al. [11] study on the effects of *E. longifolia* Jack (Tongkat Ali) alcoholic root extract against an oral pathogen. The root of *E. longifolia* ethanol extract with 200 mg/mL was tested using broth microdilution and agar disk diffusion test against *Candida albicans* and *Streptococcus mutans*. After exposure time of 24 hours on antimicrobial test, ethanol extract of *E. longifolia* root displayed a positive antibacterial effect on *S. mutans* and a positive antifungal effect on *C. albicans*. The control group drugs used in this study are nystatin and ampicillin.

Danial et al. [13] evaluated on the topic of antibacterial activity on in vivo plant parts of medicinally important *E. longifolia* (Tongkat Ali). Methanol extract with a concentration of 50 mg/mL from the roots, leaves, branches, seeds, bark, and stem core of *E. longifolia* was tested using agar disk diffusion method against *Bacillus cereus*, *Bacillus subtilis*, *Escherichia coli*, *Pseudomonas aeruginosa*, *Shigella flexneri*, and *Staphylococcus aureus*. After exposure time of 24 hours on antimicrobial test, the result indicated that the extracted compound from the root of *E. longifolia* gives the most effective antibacterial activity on *B. subtilis* (CDR), *E. coli* ATCC 25922, *P. aeruginosa* ATCC 27853, *Shigella flexneri* ATCC 12022, and *S. aureus* ATCC 25923. The control group drug used in this study is chloramphenicol.

Faisal et al. [14] study on in vitro antibacterial activity of *E. longifolia* Jack (Tongkat Ali) root extract. The ethanolic extracts of *E. longifolia*'s root with concentration of 50, 150, and 150 mg/mL were tested using agar disk diffusion method against *Bacillus cereus*, *Escherichia coli*, *Pseudomonas aeruginosa*, *Salmonella typhi*, and *Staphylococcus aureus*. The ethanolic extracts of *E. longifolia*'s root give positive results against Gram-positive (*B. cereus* and *S. aureus*) and Gram-negative bacteria (*S. typhi*). *Bacillus cereus* and *S. typhi* indicated inhibition zone values higher than the positive control values. *Escherichia coli* and *P. aeruginosa*, on the other hand, did not exhibit any signs of inhibition when tested with the ethanolic extract, classified as a negative result. The control group drugs used in this study are erythromycin and ciprofloxacin.

Faisal et al. [15] evaluated on antifungal activity of *E. longifolia* Jack (Tongkat Ali) root extract.

The ethanolic extracts of *E. longifolia*'s root with concentrations of 50, 150, and 150 mg/mL were tested using broth microdilution method and agar disk diffusion assay test against *Candida albicans* and *Aspergillus fumigatus*. The ethanolic extract of *E. longifolia* Jack root indicated positive antifungal activity against *C. albicans* and *A. fumigatus*. The control drug group used in this experiment is nystatin.

Farouk and Benafri [16] study on antimicrobial activity of *E. longifolia* Jack. The leaves, stem, and root of *E. longifolia* with different extraction solvents (methanol, ethanol, acetone, and water) at a concentration of 100 mg/mL were tested using agar disk diffusion assay method against *Bacillus subtilis*, *Escherichia coli*, *Enterococcus faecalis*, *Micrococcus luteus*, *Proteus vulgaris*, *Salmonella typhi*, *Serratia marcescens*, and *Staphylococcus aureus*. Except for two strains of Gram-negative bacteria (*Escherichia coli* and *Salmonella typhi*), the alcoholic and acetone extracts of the leaves and stem extract were active against both Gram-positive and Gram-negative bacteria. Gram-positive and Gram-negative bacteria were not inhibited by the root extract. Aqueous extract from the leaves was found to be antibacterial against *S. aureus* and *Serratia marcescens* bacteria. The control drug group of this experiment is tetracycline and chloramphenicol.

Khanam et al. [21] study on the topic of phytochemical screening and antimicrobial activity from root and stem extracts of wild *E. longifolia* Jack (Tongkat Ali). The types of extract used in this study are ethyl acetate, petroleum ether, chloroform, acetone, and methanol, which tested against *Aspergillus niger*, *B. cereus*, *E. coli*, *P. aeruginosa*, *Salmonella* Virchow, and *S. aureus* by disk diffusion assay method. Antimicrobial activity was found to be dose-dependent in all extracts. However, both stem and root extracts showed the most antibacterial activity against Gram-positive bacteria. Despite this, stem extracts were more effective against *Bacillus cereus* and *Staphylococcus aureus* than root extracts. The ethyl acetate extract from the stem indicated only moderate activity against *Pseudomonas aeruginosa*, a Gram-negative bacterium, but high activity against *Aspergillus niger*, a fungus. The control drug group used in this experiment was ampicillin.

Kuspradini et al. [23] evaluated comparative antimicrobial studies on *E. longifolia* Jack, *Rennellia elliptica* Korth, and *Trivalvaria macrophylla* Miq. against *C. albicans*, *S. aureus*, *S. mutans*, and *Streptococcus sobrinus.* The root of *E. longifolia* ethanol extract was used in agar well diffusion method. The result showed that the activity index (AI) was found in *E. longifolia* (0.96 at 1000 *μ*g concentration) that is the highest against the selected pathogens. The control drug group used in this experiment is chloramphenicol.

Lee et al. [24] stated that pasakbumin-A alone control intracellular *Mycobacterium tuberculosis* (Mtb) growth by increasing the production of neutrophils (NO) and TNF-*α* in macrophages and protecting against host cell death during Mtb infection. However, data suggested that the combination of pasakbumin-A with an anti-TB drug (rifampicin) effectively suppressed intracellular Mtb growth by promoting proinflammatory cytokine production and blocking the production of anti-inflammatory cytokine in macrophages. The root of *E. longifolia* with ethanol extract was used in this experiment and was carried out using the lactate dehydrogenase method test.

The effect of *E. longifolia* Jack extracts on salivary microorganisms such as *Streptococcus mutans*, *Lactobacillu*s, and *Candida albicans* was study by Ramzi et al. [27]. After exposure times of 72 hours in disk diffusion assay, all the microorganism tests showed positive zones of inhibition. The exhibiting zones of inhibition were 8.3 ± 0.7 mm in *S. mutans*, 12.4 ± 2.4 mm in *Lactobacillus*, and 21.4 ± 2.7 mm in *C. albicans*. These concentrations of 250 mg/mL, 125 mg/mL, 62.5 mg/mL, 31.3 mg/mL, and 0 mg/mL were used at the test microorganisms for minimum inhibitory concentration (MIC). The MIC showed that *S. mutans* was 62.5 mg/mL, *Lactobacillu*s was 125 mg/mL, and *C. albicans* was 31.3 mg/mL. An aqueous type of *E. longifolia* root extract was used in this study.

Yi Xin et al. [29] studied on the antibacterial potential of Malaysian ethnomedicinal plants against methicillin-resistant *Staphylococcus aureus* (MRSA) and methicillin-susceptible *Staphylococcus aureus* (MSSA). The leaves of *E. longifolia* methanol extract were used in the microdilution method against selected pathogen. After 22 hours of exposure to antimicrobial assay, minimum inhibitory concentration (MIC) and minimum bactericidal concentration (MBC) values showed >800 *μ*g/mL, which is considered inactive against tested microorganisms. Hence, the study proved that the leaves of *E. longifolia* methanol extract did not have an antimicrobial effect against MSSA and MRSA bacteria.

### 4.2. Effectiveness of Antiparasitic Activity of *E. longifolia*

A total of 9 in vitro studies and 1 in vivo study were evaluated on the antiparasitic activity of *E. longifolia* against 5 parasite species tested in Table 3. Based on the results, it showed that *E. longifolia* have antiparasitic activity on the entire parasite tested, in which 10 out of 10 studies showed complete positive results.  Table 5 shows the result extracted from 10 studies, which evaluate on antimicrobial activity of *E. longifolia*.

Study on antiplasmodial using the lactate dehydrogenase assay of *Plasmodium falciparum* with *E. longifolia* Jack extracts has been conducted by Chan et al. [12]. The root of *E. longifolia* ethanol, diethyl ether, and n-butanol extract with 20 mg/mL was used in this experiment. After exposure time of 72 hours on the test, quassinoids, the compounds that were isolated from the stems of *E. longifolia*, showed a positive antimalaria properties against in vitro culture of chloroquine-resistant *P. falciparum.*

Girish et al. [17] evaluated *E. longifolia* as a possible therapeutic candidate against *Blastocystis* sp. In this study, they were screened a few plant extracts. Among all the extracts, *E. longifolia* extracts showed the most antiprotozoal effect at the concentration 1.0 mg/mL. Then, they made comparison between 2 types of extraction of *E. longifolia* which is water and ethyl acetate. The ethyl acetate extraction showed a slightly higher percentage of antiprotozoal effect at 1.0 mg/mL across subtypes ST1 (94.9%), ST3 (95.1%), and ST5 (94.3%). Metronidazole (MTZ) showed the highest antiprotozoal effect across subtypes ST1 (95.8%), ST3 (93.4%), and ST5 (90.8%) when tested with allopathic drugs, at the same concentration.

Hout et al. [18] study on screening of selected indigenous plants of Cambodia for antiplasmodial activity using the root, stem, and bark of *E. longifolia*. The experiment was evaluated using the flow cytometry method against chloroquine-resistant *Plasmodium falciparum* strain. After 48 hours of exposure time to the extract, a higher antiplasmodial activity was discovered for *E. longifolia* with IC50 values of <3 mg/mL. *Eurycoma longifolia* bark, with dichloromethane, CH2Cl2 extract was the most efficient extract showing the highest antiplasmodial activity against W2.

Jiwajinda et al. [19] study on in vitro antitumour promoting and antiparasitic activities of the quassinoids from *E. longifolia* leaves. The leaves of *E. longifolia* ethanol extract with concentrations of 2, 20, and 200 mg/mL were tested against schistosomes of *Schistosoma japonicum* and chloroquine-resistant *Plasmodium falciparum* strain. The result has been evaluated using the viable cell count method. After 24 hours of exposure to the extract, when compared with those of control experiments using only dimethyl sulfoxide (DMSO), compounds 1, 3, and 5 give a significant inhibitory effect on adult schistosome movement (IM) and egg-laying (EL) of *S. japonicum* at 200 mg/mL. However, the antischistosomal effect is weaker between the three compounds as compared to the control drug at the concentration of 20 mg/mL.

Study on in vitro anti-*Toxoplasma gondii* activity of root extract of *E. longifolia* Jack was conducted by Kavitha et al. (2012). The root of *E. longifolia* methanol extract with tested against *Toxoplasma gondii.* After 36 h of exposure to the *E. longifolia* fraction, the host Vero cells showed no remarkable morphological changes and no visible intracellular parasite. TAF 355 and TAF 401 fractions showed the most efficient anti-*Toxoplasma gondii* effects. This result was indicated through a microslide tube test with a comparison of the control drug, clindamycin effect.

Kavitha et al. (2012) carried out real-time anti-*Toxoplasma gondii* activity of an active fraction of *E. longifolia* root, studied by in situ scanning and transmission electron microscopy. The result showed the significant antiparasitic activity demonstrated by the TAF355 and TAF401 active fractions of *E. longifolia*. The active fractions from *E. longifolia* designated as TAF 355 and TAF 401 have potent and selective antiproliferative activity against *T. gondii* tachyzoites.

Kuo et al. [22] study on antimalarial constituents and cytotoxic effect from the *E. longifolia* root methanol extract using biological antimalarial assays against *P. falciparum* clones, W2 and D6. The result proved that eurycomanone and pasakbumin-B compounds exhibited efficacy antimalarial activity against the resistant *P. falciparum*. Both compounds showed marginal antimalarial activity against both the W2 and D6 *P. falciparum* clones.

Mohd Ridzuan et al. [25] evaluated a study on the effect of *E. longifolia* extract on the glutathione (GSH) level in *Plasmodium falciparum*-infected erythrocytes in vitro. The study is aimed at suppressing the production of GSH in chloroquine-resistant *Plasmodium falciparum* strain to inhibit the growth of the selected pathogen. Based on the result of the study, about 95% to 100% growth inhibition of *P. falciparum*-infected erythrocyte was observed when treated with TA164 and buthionine sulfoximine (BSO), at 16 *μ*g/mL and 64 *μ*g/mL, respectively. However, TA164 fails to suppress the GSH content of enriched trophozoite-infected erythrocyte as much as BSO.

Mohd Ridzuan et al. [26] carried out an in vivo study on *E. longifolia* extract and artemisinin combination to suppress parasitemia of *Plasmodium yoelii*-infected mice. The root of *E. longifolia* methanol extract was inoculated into *Plasmodium yoelii*-infected mice before the erythrocyte of the mice being observed under microscope for viable cell count after 96 hours of exposure time to the extract. At 10 mg/kg, parasitemia of *P. yoelii*-infected mice was suppressed to 25 percent as compared to control mice, while at 30 mg/kg and 60 mg/kg, parasitemia was significantly suppressed to 41 percent and 51 percent, respectively (*p* < 0.05), using TA164. These data showed a greater effect of parasitemia suppression with TA164 compared to artemisinin drug alone.

Sriwilaijaroen et al. [28] study on antiplasmodial effects of *Brucea javanica* (L.) Merr. and *E. longifolia* Jack extracts and their combination with chloroquine and quinine on *Plasmodium falciparum* in culture. *Eurycoma longifolia* roots with aqueous, ethyl alcohol, ethyl acetate, ethanol, and methanol extracts were used against the multidrug-resistant *Plasmodium falciparum* strain K1. Ethanol and methanol extracts showed the higher activities than the other solvent extract after comparison has been made. In addition, not only quassinoid glycosides are responsible for the antimalarial activity, but the same effects were also shown in coumarins and flavonoids that were found in thin-layer chromatography.

## 5. Conclusion and Recommendations

When it comes to reviewing the data of the selected journal articles for this systematic review, we summarise that the root extracts of *E. longifolia* have the most efficient antimicrobial and antiparasitic activity compared to other plant components. *Eurycoma longifolia* can be suggested as an antimicrobial agent as broad-spectrum as it is most effective against Gram-negative, Gram-positive, and fungal species tested. *Eurycoma longifolia* can also be used as an antiparasitic agent against specific parasites tested in the selected studies.

As for the future prospect for *E. longifolia*, an in vitro study shows that roots and other plant components extracts have antimicrobial and antiparasitic properties against pathogenic microorganisms. Nevertheless, to justify and further analyse the potential of *E. longifolia* extracts as reliable antimicrobial and antiparasitic medicines, animal models are required in clinical trials. Additional research into the mechanism of action for these extracts would be advantageous to the pharmaceutical sector in order to maximise the potential of these compounds. In addition, the food industry is actively searching for other agents and natural preservatives as alternatives to synthetic compounds used in food processing, particularly for livestock consumption.

Based on the analysing results, we conclude that *E. longifolia* has an antimicrobial and antiparasitic effect, as shown to have proven against both microorganisms and parasite testing. For that reason, to prove these biological effects, more in vivo studies are needed.

## Figures and Tables

**Figure 1:** The flowchart diagram of this study (as described in the PRISMA Statement).

**Table 1:** Searching method using four main databases.

**Database** Search and/or terms
**Scopus** (“eurycoma longifolia”) AND (“antimicrobial activity”) OR (“biofilms”) OR (“antibacterial”) OR (“antifungal”) OR (“antiparasitic”)
**PubMed** **#1** Eurycoma Longifolia **#2** “antimicrobial” [MeSH terms] OR “antimicrobial” OR “Agents, Anti-Infective” OR “Anti Infective Agents” OR “Antiinfective Agents” OR “Agents, Antiinfective” OR “Microbicides” OR “Antimicrobial Agents” OR “Agents, Antimicrobial” OR “Anti-Microbial Agents” OR “Agents, Anti-Microbial” OR “Anti-Microbial Agents” **#3** “biofilms” [MeSH terms] OR “biofilms” OR “Bacterial Adhesion” OR “Adhesins, Bacterial” OR “Biofouling” **#4** “antibacterial” [MeSH terms] OR “antibacterial” OR “Agents, Anti-Bacterial” OR “Anti-Bacterial Agents” OR “Antibacterial Agents” OR “Agents, Antibacterial” OR “Antibiotics” OR “Bacteriocidal Agents” OR “Agents, Bacteriocidal” OR “Bacteriocides” OR “Anti-Mycobacterial Agents” OR “Agents, Anti-Mycobacterial” OR “Anti Mycobacterial Agents” OR “Antimycobacterial Agents” OR “Agents, Antimycobacterial” **#5** “antifungal” [MeSH terms] OR “antifungal” OR “Agents, Antifungal” OR “Therapeutic Fungicides” OR “Fungicides, Therapeutic” OR “Antibiotics, Antifungal” OR “Antifungal Antibiotics” **#6** “anti-parasitic” [MeSH terms] OR “anti-parasitic” OR “Agents, Anti-parasitic” OR “Anti-parasitic Drugs” OR “Drugs, Antiparasitic” OR “Parasiticides” OR “Antiparasitics” **#2 OR #3 OR #4 OR #5 OR #6 AND #1**
**ScienceDirect** “eurycoma longifolia” AND “antimicrobial”
**Google Scholar** Search manually from previous studies.

**Table 2:** Characteristics of the included articles.

Study	Assay	Microorganism tested	Plant parts	Types of extract	Antimicrobial assay	Exposure times in the antimicrobial test	Control groups	Sample size	Main results
[11]	Effects of *Eurycoma Longifolia* Jack (Tongkat Ali) alcoholic root extract against oral pathogens	*Candida albicans* and *Streptococcus mutans*	Root	Ethanol	Agar disk diffusion and broth microdilution test	24 h	Nystatin, ampicillin	*n* = 3	Ethanol extracts of *E. longifolia* Jack root displayed a positive antibacterial effect on *S. mutans* and a positive antifungal effect on *C. albicans*
[12]	Antiplasmodial studies of *Eurycoma longifolia* Jack using the lactate dehydrogenase assay of *Plasmodium falciparum*	*Plasmodium falciparum*	Root	Ethanol, diethyl ether and *n*-butanol	Lactate dehydrogenase method	72 h	Untreated medium	*n* = 3	Quassinoids isolated from *E. longifolia* showed potential antimalarial properties against in vitro culture of chloroquine-resistant *P. falciparum*
[13]	Antibacterial studies on in vivo plant parts of medicinally important *Eurycoma longifolia* (Tongkat Ali)	*Escherichia coli*, *Pseudomonas aeruginosa*, *Bacillus cereus*, *Staphylococcus aureus*, *Shigella flexneri*, and *Bacillus subtilis*	Roots, leaves, branches, seeds, bark, and stem core	Methanol	Agar disk diffusion assay	24 h	Chloramphenicol	*n* = 3	The result indicated that the most effective antibacterial agent is the extracted compound from the roots of *Eurycoma longifolia* on *Escherichia coli* ATCC 25922, *Pseudomonas aeruginosa* ATCC 27853, *Bacillus subtilis* (CDR), *Staphylococcus aureus* ATCC 25923, and *Shigella flexneri* ATCC 12022.
[14]	In vitro antibacterial activity of *Eurycoma longifolia* Jack (Tongkat Ali) root extract	*Bacillus cereus, Staphylococcus aureus, Pseudomonas aeruginosa, Escherichia coli* and *Salmonella typhi*	Root	Ethanol	Agar disk diffusion and broth microdilution test	24 h	Erythromycin and ciprofloxacin	*n* = 3	The ethanolic extract of *E. longifolia* Jack root extract showed positive results against Gram-positive bacteria (*S. aureus* and *B. cereus*) and Gram-negative (*S. typhi*). *B. cereus* and *S. typhi* showed inhibition zone values higher than the positive control values. However, *E. coli* and *P. aeruginosa* did not show any inhibition by the ethanol-based extract.
[15]	Antifungal activity of *Eurycoma longifolia* jack (Tongkat Ali) root extract	*Candida albicans* and *Aspergillus fumigatus*	Root	Ethanol	Agar disk diffusion assay and broth microdilution method test	48 h	Nystatin	*n* = 3	The ethanolic extract of *E. longifolia* Jack root showed positive antifungal activity against *C. albicans* and *A. fumigatus*
[16]	Antibacterial activity of *Eurycoma longifolia* Jack: a Malaysian medicinal plant	*Bacillus subtilis*, *Staphylococcus aureus*, *Enterococcus faecalis*, *Micrococcus luteus*, *Escherichia coli*, *salmonella typhi*, *Proteus vulgaris*, and *Serratia marcescens*	Leaves, stem, and root	Methanol, ethanol, acetone and water	Agar well diffusion method	24 h	Tetracycline and chloramphenicol	*n* = 3	The alcoholic and acetone extracts of the leaves and stem extracts were active on both Gram-positive and Gram-negative bacteria except against 2 strains of Gram-negative bacteria (*Escherichia coli* and *salmonella typhi*). The root extracts had no antibacterial activity against Gram-positive and Gram-negative bacteria tested. Aqueous leaf extract showed antibacterial activity against *Staphylococcus aureus* and *Serratia marcescens.*
[17]	Tongkat Ali (*Eurycoma longifolia*): a possible therapeutic candidate against *Blastocystis* sp.	*Blastocystis* sp.	Roots	Crude aqueous, ethyl acetate, and water	Viable cell count	72 h	Untreated medium	*n* = 3	Based on the screening process, among all the extracts, Tongkat Ali exhibited the highest antiprotozoal activity at 1.0 mg/mL. Between the water and ethyl acetate fractions of Tongkat Ali, the ethyl acetate fraction exhibited a slightly higher percentage of antiprotozoal activity at 1.0 mg/mL across subtypes ST1 (94.9%), ST3 (95.1%), and ST5 (94.3%). When tested with allopathic drugs at the same concentration, MTZ exhibited the highest antiprotozoal activity across subtypes ST1 (95.8%), ST3 (93.4%), and ST5 (90.8%).
[18]	Screening of selected indigenous plants of Cambodia for antiplasmodial activity	Chloroquine-resistant *Plasmodium falciparum* strain	Roots, stem, and bark	Aqueous, methanol and dichloromethane	Flow cytometry	48 h	Chloroquine	*n* = 3	A very high antiplasmodial activity was observed for *E. longifolia* with IC50 values of <3 mg/mL. Tongkat Ali bark with CH2Cl2 is the most efficient extract showing the most increased antiplasmodial activity against W2.
[19]	In vitro antitumour promoting and antiparasitic activities of the quassinoids from *Eurycoma longifolia*, a medicinal plant in Southeast Asia	Schistosomes of *Schistosoma japonicum* and chloroquine-resistant *Plasmodium falciparum* strain	Leaves (quassinoids)	Ethanol	Viable cell count	24 h	Praziquantel	*n* = 3	Compounds 1, 3, and 5 showed significantly inhibitory effects on adult schistosome movement (IM) and egg-laying (EL) of *S. japonicum* at 200 mg/mL as compared with those of control experiments using only DMSO. However, the antischistosomal effect is weaker between the three compounds as compared to the control drug at the concentration of 20 mg/mL.
(Kavitha, Noordin, Chan, et al., 2012)	In vitro anti-*Toxoplasma gondii* activity of root extract/fractions of *Eurycoma longifolia* Jack	*Toxoplasma gondii*	Root	Methanol	Micro slide tubes test	24 h	Clindamycin	*n* = 3	After 36 h of exposure to the *E. longifolia* fraction, the host Vero cells showed no visible intracellular parasite and no remarkable morphological changes. TAF 355 and TAF 401 fractions are the most efficient anti-*Toxoplasma gondii* effects.
[20]	Real-time anti-*Toxoplasma gondii* activity of an active fraction of *Eurycoma longifolia* root studied by in situ scanning and transmission electron microscopy	*Toxoplasma gondii*	Root	Methanol	Electron microscopy observation	36 h	Clindamycin	*n* = 3	The significant antiparasitic activity shown by the TAF355 and TAF401 active fractions of *E. longifolia.* The active fractions from *E. longifolia* designated as TAF 355 and TAF 401 have potent and selective antiproliferative activity against *T. gondii* tachyzoites.
[21]	Phytochemical screening and antimicrobial activity of root and stem extracts of wild *Eurycoma longifolia* Jack (Tongkat Ali)	*A. niger*, *Escherichia coli*, *Salmonella* Virchow, *P. aeruginosa*, *B. cereus*, and *S. aureus*	Root and stem	Petroleum ether, chloroform, ethyl acetate, acetone and methanol	Disk diffusion assay	24 h	Ampicillin	*n* = 3	All the extracts exhibited dose-dependent antimicrobial activity. However, the highest antibacterial activity was observed against Gram-positive bacteria by both stem and root extracts. Nevertheless, stem extracts were more potent than root extracts against *Bacillus cereus* and *Staphylococcus aureus*. Merely, ethyl acetate extract of the stem showed moderate activity against Gram-negative bacteria, *Pseudomonas aeruginosa*, and high activity against fungus, *Aspergillus niger.*
[22]	Cytotoxic and antimalarial constituents from the roots of *Eurycoma longifolia*	*P. falciparum* clones W2 and D6		Methanol	Biological antimalarial assays	Not stated	Mefloquine and chroquine	*n* = 3	Compounds 57 and 58 displayed potent antimalarial activity against the resistant *Plasmodium falciparum*. Eurycomanone (57) and pasakbumin-B (58) exhibited marginal antimalarial activity against both the W2 and D6 *P. falciparum* clones.
[23]	Comparative antimicrobial studies on plant species known as “pasak bumi': *Eurycoma longifolia* Jack, *Rennelia elliptica* Korth. And *Trivalvaria macrophylla* Miq. (version 1; peer review: 1 approved, 1 approved with reservations)	*Candida albicans*, *Staphylococcus aureus*, *Streptococcus mutans*, and *streptococcus sobrinus*	Root	Ethanol	Agar well diffusion method	24 h	Chloramphenicol	*n* = 3	The highest activity index (AI) was found in the *E. longifolia* (0.96 at 1000 *μ*g concentration) against selected pathogens.
[24]	Pasakbumin-A controls the growth of *mycobacterium tuberculosis* by enhancing the autophagy and production of antibacterial mediators in mouse macrophages	*Mycobacterium tuberculosis*		Water	Lactate dehydrogenase method	72 h	Rifampicin	*n* = 3	Pasakbumin-A alone controls intracellular Mtb growth by enhancing the production of NO and TNF-*α* in macrophages and protects against host cell death during Mtb infection. However, data suggested that the combination of pasakbumin-A with an anti-TB drug (rifampicin) effectively suppressed intracellular Mtb growth by promoting the production of proinflammatory cytokine and blocking the production of anti-inflammatory cytokine in macrophages.
[25]	Effect of *Eurycoma longifolia* extracts on the glutathione level in *plasmodium falciparum*-infected erythrocytes in vitro.	Chloroquine-resistant *Plasmodium falciparum* strain	Root	Methanol	Growth inhibition assay	36 h	Untreated medium	*n* = 3	About 95% to 100% growth inhibition of *P. falciparum*-infected erythrocyte was observed when treated with TA164 and BSO at 16 *μ*g/mL and 64 *μ*g/ml, respectively. TA164 fails to suppress the GSH content of enriched trophozoite-infected erythrocyte as much as buthionine sulphoximine.
[26]	*Eurycoma longifolia* extract-artemisinin combination: parasitemia suppression of *Plasmodium yoelii*-infected mice.	*Plasmodium yoelii*	Root	Methanol	Viable cell count	96 h	Artemisinin	*n* = 5	At 10 mg/kg, parasitemia of *P. yoelii-*infected mice was suppressed to 25 percent as compared to control mice, while at 30 mg/kg and 60 mg/kg, parasitemia was significantly suppressed to 41 percent and 51 percent, respectively (*p* < 0.05) using TA164. These data showed a more significant effect of parasitemia suppression with TA164 than with artemisinin drug alone.
[27]	The effect of *Eurycoma longifolia* Jack (Tongkat Ali) root extract on salivary *S. mutans*, *lactobacillus* and *Candida albicans* isolated from high-risk caries adult patients	*S. mutans*, *Lactobacillus*, and *Candida albicans*	Root	Ethanol	Disk diffusion assay and broth dilution method	72 h	Chlorhexidine, ampicillin and nystatin	*n* = 9	Disk diffusion assay showed positive zones of inhibition for all test microorganisms with *S. mutans*, *Lactobacillus*, and *C. albicans* exhibiting zones of inhibition of 8.3 ± 0.7 mm, 12.4 ± 2.4 mm, and 21.4 ± 2.7 mm, respectively. For minimum inhibitory concentration, the test microorganisms were tested at concentration of 250 mg/mL, 125 mg/mL, 62.5 mg/mL, 31.3 mg/mL, and 0 mg/mL. The minimum inhibitory concentration showed that MIC of *S. mutans* was at 62.5 mg/mL, *Lactobacillus* at 125 mg/mL, and *C. albicans* at 31.3 mg/mL.
[28]	Antiplasmodial effects of *Brucea javanica* (L.) Merr. and *Eurycoma longifolia* jack extracts and their combination with chloroquine and quinine on *Plasmodium falciparum* in culture	*Plasmodium falciparum*	Root	Methanol-ethanol, ethanol, ethyl acetate, ethyl alcohol, and distilled water	Checkerboard technique	24 h	Chloroquine and quinine	*n* = 3	Antiplasmodial activity of *E. longifolia* with methanol-ethanol extract showed higher activities than the other solvent extract after comparison has been made.
[29]	Antibacterial potential of Malaysian ethnomedicinal plants against methicillin-susceptible *Staphylococcus aureus* (MSSA) and methicillin-resistant *Staphylococcus aureus* (MRSA)	Methicillin-resistant *Staphylococcus aureus* (MRSA) and methicillin-sensitive *Staphylococcus aureus* (MSSA)	Leaves	Methanol	Microdilution method	22 h	Vancomycin and ciprofloxacin	*n* = 3	MIC and MBC values showed >800 mg/mL, which is considered inactive against tested microorganisms.

**Table 3:** Selected microorganism species.

Gram-positive bacteria	Gram-negative bacteria	Fungi	Parasite
(i) *Strep. mutans* (ii) *Bacillus cereus* (iii) *Staph. aureus* (MRSA, MSSA) (iv) *Bacillus subtilis* (v) *Enterococcus faecalis* (vi) *Strep. sobrinus* (vii) *Lactobacillus* (viii) *Mycobacterium tuberculosis*	(i) *E. coli* (ii) *Pseudomonas aeruginosa* (iii) *Shigella flexneri* (iv) *Proteus vulgaris* (v) *Serratia marcescens* (vi) *Salmonella* Virchow (vii) *Salmonella typhi*	(i) *Candida albicans* (ii) *Aspergillus fumigatus* (iii) *Aspergillus niger*	(i) *Plasmodium falciparum* (chloroquine-resistant) (ii) *Blastocystis* spp. (iii) *Toxoplasma gondii* (iv) *Toxoplasma yoelii*

**Table 4:** Results for selected studies of antimicrobial activity of *Eurycoma longifolia.*

Studies	Plant components	Positive result	Negative result
[11]	Root	*Candida albicans* and *Streptococcus mutans*	—
[13]	Roots, leaves, branches, seeds, bark, and stem core	*Escherichia coli*, *Pseudomonas aeruginosa*, *Bacillus cereus*, *Staphylococcus aureus*, *Shigella flexneri*, and *Bacillus subtilis*	—
[14]	Root	*Bacillus cereus*, *Staphylococcus aureus*, and *Salmonella typhi*	*Pseudomonas aeruginosa*, *Escherichia coli*
[15]	Root	*Candida albicans* and *Aspergillus fumigatus*	—
[16]	Leaves, stem, and root	*Bacillus subtilis*, *Staphylococcus aureus*, *Enterococcus faecalis*, *Micrococcus luteus*, *Proteus vulgaris*, and *Serratia marcescens*	*Escherichia coli*, *Salmonella typhi*
[21]	Root and stem	*A. niger*, *Escherichia coli*, *Salmonella* Virchow, *P. aeruginosa*, *B. cereus*, and *S. aureus*	—
[23]	Root	*Candida albicans*, *Staphylococcus aureus*, *Streptococcus mutans*, and *Streptococcus sobrinus*	—
[24]	Root	*Mycobacterium tuberculosis*	—
[27]	Root	*S. mutans*, *Lactobacillus*, and *Candida albicans*	—
[29]	Leaves	—	Methicillin-resistant *Staphylococcus aureus* (MRSA) and methicillin-sensitive *Staphylococcus aureus* (MSSA)

**Table 5:** Results for selected studies of antimicrobial activity of *Eurycoma longifolia.*

Studies	Plant components	Positive result	Negative result
[12]	Root	*Plasmodium falciparum*	—
[17]	Root	*Blastocystis* sp.	—
[18]	Root, stem, and bark	Chloroquine-resistant *Plasmodium falciparum* strain	—
[19]	Leaves	Schistosomes of *Schistosoma japonicum* and chloroquine-resistant *Plasmodium falciparum* strain	—
[30]	Root	*Toxoplasma gondii*	—
[20]	Root	*Toxoplasma gondii*	—
[22]	Root	*P. falciparum* clones W2 and D6	—
[25]	Root	Chloroquine-resistant *Plasmodium falciparum* strain	—
[26]	Root	*Plasmodium yoelii*	—
[28]	Root	*Plasmodium falciparum*	—

## Data Availability

The data are made available upon request.
